The article "The Value of CT Perfusion Parameters and Apparent Diffusion Coefficient Value of Magnetic Resonance Diffusion Weighted Imaging in Diagnosis of Hepatocellular Carcinoma" was retracted in 2023. Reasons: signs of a paper mill; compromised peer review; unreliable results or conclusions.

# The Value of CT Perfusion Parameters and Apparent Diffusion Coefficient Value of Magnetic Resonance Diffusion Weighted Imaging in Diagnosis of Hepatocellular Carcinoma

**DOI:** 10.1155/2022/2771869

**Published:** 2022-09-27

**Authors:** Kezhen Li, Baiping Wang

**Affiliations:** ^1^Medical Imaging Department, Wanning People's Hospital, 571500, China; ^2^Department of Radiology, The Second Affiliated Hospital of Hainan Medical University, 570311, China

## Abstract

**Background:**

Hepatocellular carcinoma is one of the malignant tumors with the highest incidence in the world. According to the latest statistics of the National Cancer Center, the incidence of liver cancer ranks fifth in malignant tumors and its mortality rate ranks second in China, which seriously threatens people' s life and health.

**Aim:**

To investigate the value of CT perfusion parameters and apparent diffusion coefficient (ADC) of magnetic resonance imaging (MRI) diffusion weighted imaging (DWI) in the diagnosis of hepatocellular carcinoma.

**Methods:**

43 patients with hepatocellular carcinoma and 40 patients with hepatic hemangioma treated in our hospital from August 2018 to August 2021 were selected for CT perfusion imaging and MRI examination.

**Results:**

The liver blood flow (BF), liver blood volume (BV), and hepatic artery perfusion (HAP) in the hepatocellular carcinoma group were (267.38 ± 35.59) ml/(min·100 g), (30.20 ± 8.82) ml/100 g, and (0.64 ± 0.10) ml/(min·ml), respectively, which were significantly higher than those in the hepatic hemangioma group (*p* < 0.05). The ADC value of hepatocellular carcinoma DWI sequence was (1.20 ± 0.17) ×10^−3^ mm^2^, which was significantly lower than that of hepatic hemangioma (*p* < 0.05). The area under ROC curve of BF, BV, HAP, and ADC values for hepatocellular carcinoma was 0.860, 0.754, 0.804, and 0.890, respectively. The area under ROC curve of the four groups was compared (*p* > 0.05).

**Conclusion:**

CT perfusion parameters BF, BV, HAP, and DWI sequence ADC values have certain application value in the diagnosis of hepatocellular carcinoma, and there is no significant difference between the diagnostic value of each parameter.

## 1. Introduction

Hepatocellular carcinoma is the most common malignant tumor in China, with the characteristics of occult onset and rapid progress [1, 2]. There is no special symptom in the early stage of liver cancer, and patients often present with pain in the liver area, anorexia, and dyspepsia. When there is a serious symptom, most patients have reached the advanced stage of cancer. At this time, retreatment can only prolong the survival time of patients and cannot cure the disease [3, 4]. Therefore, the early diagnosis of hepatocellular carcinoma is of great importance, and CT and magnetic resonance imaging (MRI) are commonly used [5, 6]. However, the soft tissue density resolution of CT is poor, and the detection rate and qualitative of lesions are also insufficient. Relevant studies have found that hepatocellular carcinoma can cause abnormal blood flow in the portal vein of the body. CT perfusion imaging can detect the above changes, so CT perfusion imaging has a certain diagnostic effect on hepatocellular carcinoma [7, 8]. Diffusion weighted imaging (DWI) of MRI can respond to the physiological and pathological characteristics of the body by means of the movement of water molecules in the tissue, and the most important indicator is the apparent diffusion coefficient (ADC) value [9, 10]. DWI provides a variety of analytical methods, such as DWI images, ADC maps, and ADC values, which can reflect the internal changes of malignant tumors at the cellular and molecular levels, and has unparalleled advantages in noninvasive evaluation of early tumor efficacy [11, 12]. DWI is the best method for quantitative study of microvascular perfusion and diffusion in vivo and has been successfully applied to the central nervous system [13, 14]. DWI has been gradually used for the diagnosis of abdominal disease. In liver disease, it is mainly used for the identification of lesions and the judgment of benign and malignant lesions in the early stage [15, 16]. This study aims to explore the value of CT perfusion parameters and MRI-DWI ADC in the diagnosis of hepatocellular carcinoma.

Core tips: ADC value is the most important indicator in DWI of MRI. ADC value can quantitatively analyze the benign and malignant tumors. CT perfusion imaging has a certain diagnostic effect on hepatocellular carcinoma. This study attempts to combine CT perfusion parameters and ADC values of MRI-DWI to explore its role in the diagnosis of hepatocellular carcinoma, which has certain clinical significance.

## 2. Materials and Methods

### 2.1. General Information

43 cases of hepatocellular carcinoma (HCC) and 40 cases of hepatic hemangioma treated in our hospital from August 2018 to August 2021 were selected as research subjects. Inclusion criteria: (1) All patients were confirmed by pathology. (2) Age>18 years. (3) CT and MRI examination in our hospital. (4) The clinical image data were preserved completely. (5) Informed consent has been obtained from patients and their families. Exclusion criteria: (1) A history of radiotherapy and chemotherapy before examination. (2) Patients with other systemic malignant tumors. (3) Patients who dropped out of the study. The general data of patients with hepatocellular carcinoma and hepatic hemangioma are compared in Table 1. This study has been approved by the Ethics Committee.

### 2.2. CT Perfusion Imaging

All patients underwent CT perfusion imaging. After fasting for 8 hours, the patients were assisted to take supine position with advanced feet and arms up. The sternal handle and the midpoint of the sisal process were positioned to guide the patients to carry out correct scanning breathing training. GE company 64-slice spiral CT machine was used for dynamic perfusion scanning. Scanning parameter settings: tube voltage is 120kV, tube current is 200mA, layer thickness is 1.0 mm, scanning pitch is 1.2 mm, scanning thickness is 5mm, the instrument with CT scan and enhanced scan function. Patients were given 800~1000 ml warm boiled water before examination. First of all, the upper abdomen was scanned horizontally. The larger tumor area was taken as the scanning center, and the similar layer near the lesion center was selected as the perfusion level. The scanning range was from the sternocleidomastoid to the iliac spin. The arterial phase (27 s), portal venous phase (66 s), and delayed phase (180 s) were scanned (Figure 1). The conventional CT scan was performed first, and then the CT enhanced scan mode was switched to obtain the duration and enhancement degree of the lesion, and the blood supply characteristics and internal structure of the lesion were analyzed. The contrast agent was iodixanol (BayerAGt, J20171008, Batch No. KT09T6p). The high-pressure syringe was used to inject at a rate of 4 ml/s at a dose of 1.5 ml/kg, and the scanning was delayed by 150–180 s. The data was transmitted to the SunUltraAW4 workstation. The software for processing the data was Perfusion3, and the corresponding time density curve was obtained by computer processing. After computer calculation, the blood flow (BF), blood volume (BV), hepatic arterial perfusion (HAP), and mean transit time (MTT) were obtained.

### 2.3. MRI Examination

The instrument used was SIGNACONTOUR015T MRI produced by GE Company in the United States. The patients have fasted within 4–6 h before examination, and all metal objects were removed. The coils used matched phased array coils and abdominal phased array coils. The field intensity was set to 45 mT/m, the thickness of the layer was set to 10 mm, and the layer spacing was 210 mm. The range was from the top of the diaphragm to the lower pole of the right kidney, and the respiratory gating was placed. T2 weighted imaging (T2WI), dual-echo T1 weighted imaging (T1WI), DWI, and ADC3 phase enhancement scanning were performed on the diaphragm on the abdominal transverse axis, breath holding on the transverse axis, free breathing transverse axis, and breath holding transverse axis, respectively (Figure 2). Gd-DTPA was used as the contrast agent. The injection volume was 0.1 ml/kg and the injection rate was 1.5 ml/s. The axial artery phase (26 s), portal vein phase (60s), and equilibrium phase (180 s) were scanned. Parameter settings are as follows: (1) T2WI: TR2200ms, average times 1, layer spacing 1 mm, layer thickness 5 mm, FOV 40 cm ×40 cm, matrix 252 × 213; (2) T1WI: TR3.6 ms, average times 1, layer spacing 1mm, layer thickness 5mm, FOV 40cm ×40 cm, matrix 252 × 213; (3) DWI: diffusion sensitive gradient field parameters (*b* value) were 0, 50, 400, 800 mm2/s, NSA1, layer spacing 1mm, layer thickness 5mm, FOV 40cm ×40 cm, matrix 252 × 213.

### 2.4. Statistical Processing

SPSS22.0 software was used for data analysis. Age, ADC value, and other data were expressed as (*χ* ± *s*), and *t* test was used to analyze the difference between groups. Comparison of gender and other data using 2 tests; the diagnostic value was analyzed by receiver operating characteristic (ROC) curve. *p* < 0.05 was statistically significant.

## 3. Results

### 3.1. Comparison of CT Perfusion Parameters between Hepatocellular Carcinoma and Hepatic Hemangioma

BF, BV, and HAP in hepatocellular carcinoma were significantly higher than those in hepatic hemangioma (*p* < 0.05) (see Table 2).

### 3.2. Comparison of CT Perfusion Parameters in Patients with Hepatocellular Carcinoma of Different Genders and Ages

The BF, BV, HAP, and MTT were compared between male and female patients with hepatocellular carcinoma, patients with hepatocellular carcinoma aged <50 years and ≥50 years, and patients with hepatocellular carcinoma with and without hypertension and diabetes mellitus (see Table 3).

### 3.3. Comparison of ADC Values of DWI Sequences between Hepatocellular Carcinoma and Hepatic Hemangioma

ADC value of hepatocellular carcinoma DWI sequence was significantly lower than that of hepatic hemangioma (*p* < 0.05) (see Table 4).

### 3.4. Comparison of ADC Values of DWI Sequences in Patients with Hepatocellular Carcinoma of Different Genders and Ages

DWI ADC values were compared between male and female patients with hepatocellular carcinoma, patients with hepatocellular carcinoma aged <50 years and ≥50 years, and patients with hepatocellular carcinoma with and without hypertension and diabetes mellitus (see Table 5).

### 3.5. Judgmental Value

The areas under ROC curves of BF, BV, HAP, and ADC values for HCC were 0.860, 0.754, 0.804, and 0.890, respectively, *p* < 0.05, and the areas under ROC curves of the four were compared (*p* > 0.05). The specific parameters are shown in Table 6 and Figure 3.

## 4. Discussion

Most people believe that the etiology of hepatocellular carcinoma is closely related to viral infection and environmental factors [17, 18] However, the initial symptoms are not obvious, bringing great difficulties to clinical diagnosis and treatment. Effective diagnosis is an important prerequisite for formulating treatment measures and evaluating curative effect. Therefore, it is particularly necessary to conduct timely, accurate, and effective examinations and study the patient ‘s disease-related indicators [19, 20].

According to relevant research reports [21, 22], the accuracy of CT examination of liver cancer is very high, and the diagnostic value of small lesions is also very high. Therefore, the clinical acceptance of CT examination is very high, and CT examination has become the most commonly used method for the diagnosis of primary liver cancer. At the same time, as the blood flow of malignant tumor patients is mostly obviously abnormal, CT perfusion imaging can clearly display the anatomical details of small lesions and hepatocellular carcinoma, and reflect the blood flow.

The results showed that there was no significant difference in BF, BV, HAP, and MTT between male and female patients with hepatocellular carcinoma and patients aged <50 and ≥50 years old. It suggested that different ages and genders did not affect factors such as liver blood flow. The results of this study showed that BF, BV, and HAP in HCC group were significantly higher than those in hepatic hemangioma group. After the patient developed into hepatocellular carcinoma, the blood perfusion status of the liver changed to a certain extent. With the malignant proliferation of cancer, the blood flow in the artery becomes larger, which leads to insufficient blood supply in the portal vein. Therefore, the judgment of the nature of the tumor can also be reflected by the supply of arterial blood. In the detection of new blood vessels in liver cancer cells, the flow rate is accelerated, resulting in a certain degree of damage to vascular endothelial cells. Due to the presence of different sizes of arteries and veins, arterial portal vein and other different ways and levels of direct entry into the tumor, BV, BF, and HAP increased.

The results of this study showed that there was no significant difference in ADC values of DWI sequences between male and female patients with hepatocellular carcinoma, age <50 years and age ≥50 years. After excluding the influence of age and gender on ADC, it was found that the ADC value of hepatocellular carcinoma DWI sequence was significantly lower than that of hepatic hemangioma. The reason is that although the dispersion of water molecules is different, the b0 image signal of hepatic hemangioma is still very high, so due to T2 transmission effect, their DWI shows high signal. It has been found in some studies [23, 24] that DWI examination technology plays an increasingly important role in the identification of benign and malignant liver tumors. Due to a variety of components in tumor cells, intercellular space becomes smaller, and the diffusion of water molecules in malignant tumors is more difficult than that in normal cases, and the ADC value is also smaller than that in normal tissues. However, in the benign lesion of hemangioma, hepatic hemangioma is mainly composed of liquid components. The components in cells have little effect on the movement of water molecules, and the ADC value is larger than that of normal tissues. DWI sequence quantitatively analyzed the movement of water molecules in tissues by ADC values. DWI can detect the direction of cell permeability, capillary perfusion, and cell membrane permeability [25, 26].

MRI DWI can reflect the nature of the lesion at the histological level. For example, focal nodular hyperplasia contains normal phagocytotic hepatocytes, and the uptake of contrast agents in the process of hepatobiliary enhancement will present a slightly higher or equal signal, while hepatocellular carcinoma will not [27–29]. In normal liver cells, contrast agent uptake rate will reduce the majority of low signal, while there are still a few lesions showing high signal or equal signal. The results showed that there was no significant difference between the area under the ROC curve of liver cells and BF, BV, HAP, and ADC values. It is suggested that CT perfusion parameters BF, BV, HAP, and DWI sequence ADC values had certain value in the diagnosis of hepatocellular carcinoma and had certain application value. Although the number of cases is small, the increased specific value is not accurate, but the overall detection efficiency is certainly improved. The specific reason is that two imaging examinations can make up for each other' s shortcomings. Considering that the two methods can clearly show the solid part of the tumor and provide help for judgment, they can be used together.

There are few studies on DWI in differentiating hepatocellular carcinoma from hepatic hemangioma [30, 31]. According to this study, we found that the ADC value of DWI sequence could be used for the diagnosis of hepatocellular carcinoma, which had clinical reference significance. However, this study still has many limitations, such as the limited number of samples, which will affect statistical results. In addition, this study is limited to two types of tumors, which need to be further explored in the next study.

## 5. Conclusion

CT perfusion parameters BF, BV, HAP, and DWI sequence ADC values have certain application value in the diagnosis of hepatocellular carcinoma, and there is no significant difference between the diagnostic value of each parameter.

## Figures and Tables

**Figure 1:** CT image of hepatocellular carcinoma. (a: plain scan period; b: arterial phase; c: portal venous phase; d: delayed phase).

**Figure 2:** MRI image of hepatocellular carcinoma. (a: T2WI; b: T1WI; c: DWI; d: ADC).

**Figure 3:** ROC curve analysis.

**Table 1:** Comparison of general data of patients with hepatocellular carcinoma and hepatic hemangioma.

Group	Cases	Male/female	Age (year)	Hypertension (%)	Diabetes (%)
Hepatocellular carcinoma	43	23/20	55.60 ± 7.82	13 (30.23)	11 (25.58)
Hepatic hemangioma	40	28/12	53.49 ± 8.43	12 (30.00)	10 (25.00)
*t*/*χ*^2^		2.385	1.183	0.001	0.004
*p*		0.123	0.240	0.982	0.951

**Table 2:** Comparison of CT perfusion parameters between hepatocellular carcinoma and hepatic hemangioma.

Group	Cases	BF [ml/(min·100 g)]	BV (ml/100 g)	HAP [ml/(min·ml)]	MTT (s)
Hepatocellular carcinoma	43	267.38 ± 35.59	30.20 ± 8.82	0.64 ± 0.10	11.78 ± 1.43
Hepatic hemangioma	40	190.92 ± 31.19	21.10 ± 9.10	0.44 ± 0.12	12.03 ± 1.56
*t*		10.376	4.625	8.270	-0.762
*p*		<0.001	<0.001	<0.001	0.448

**Table 3:** Comparison of CT perfusion parameters in patients with hepatocellular carcinoma of different gender and age.

Group	Cases	BF [ml/(min·100 g)]	BV (ml/100 g)	HAP [ml/(min·ml)]	MTT (s)
Sex					
Male	23	264.40 ± 39.12	28.83 ± 6.50	0.63 ± 0.12	11.73 ± 1.55
Female	20	270.12 ± 37.10	31.10 ± 7.43	0.66 ± 0.13	11.98 ± 1.62
*t*		-0.490	-1.069	-0.787	-0.517
*p*		0.627	0.291	0.436	0.608
Age					
<50 year	24	263.39 ± 40.40	28.95 ± 5.84	0.62 ± 0.14	11.80 ± 1.62
≥50 year	19	271.11 ± 38.83	30.92 ± 6.11	0.67 ± 0.16	12.01 ± 1.70
*t*		-0.633	-1.076	-1.092	-0.413
*p*		0.530	0.288	0.281	0.682
Hypertension					
Yes	13	265.59 ± 39.29	29.01 ± 6.10	0.64 ± 0.13	11.92 ± 1.72
No	30	270.02 ± 40.11	31.01 ± 5.28	0.66 ± 0.18	12.06 ± 1.80
*t*		-0.335	-1.089	-0.361	-0.237
*p*		0.740	0.283	0.720	0.814
Diabetes					
Yes	11	267.10 ± 40.10	29.88 ± 5.98	0.65 ± 0.14	11.97 ± 1.81
No	32	271.12 ± 41.17	30.82 ± 6.12	0.67 ± 0.16	12.12 ± 1.92
*t*		-0.281	-0.442	-0.368	-0.227
*p*		0.780	0.661	0.715	0.822

**Table 4:** Comparison of ADC values of DWI sequence between hepatocellular carcinoma and hepatic hemangioma.

Group	Cases	ADC (×10^−3^ mm^2^)	*t*	*p*
Hepatocellular carcinoma	43	1.20 ± 0.17	-12.526	<0.001
Hepatic hemangioma	40	1.63 ± 0.14		

**Table 5:** Comparison of ADC values of DWI sequence in patients with hepatocellular carcinoma of different gender and age.

Group	Cases	ADC (×10^−3^ mm^2^)	*t*	*p*
Sex				
Male	23	1.18 ± 0.12	-1.177	0.246
Female	20	1.22 ± 0.10		
Age				
<50 year	24	1.19 ± 0.11	-0.467	0.643
≥50 year	19	1.21 ± 0.17		
Hypertension				
Yes	13	1.20 ± 0.13	-0.777	0.441
No	30	1.23 ± 0.11		
Diabetes				
Yes	11	1.18 ± 0.14	-1.163	0.252
No	32	1.24 ± 0.15		

**Table 6:** ROC curve parameters.

Index	Area under curve	*p*	Truncation value	Sensitivity (%)	Specificity (%)
BF	0.860	<0.001	240 ml/(min·100 g)	78.90	72.20
BV	0.754	<0.001	28.50 ml/100 g	70.40	69.00
HAP	0.804	<0.001	0.56 ml/(min·ml)	76.50	70.00
ADC	0.890	<0.001	1.30 ×10-3 mm2	84.50	78.80

## Data Availability

The datasets used and analyzed during the current study are available from the corresponding author upon reasonable request.
